The article "κ-Opioid Receptor Agonist Ameliorates Postoperative Neurocognitive Disorder by Activating the Ca2+/CaMKII/CREB Pathway" was retracted in 2022. Reason: compromised peer review.

# *κ*-Opioid Receptor Agonist Ameliorates Postoperative Neurocognitive Disorder by Activating the Ca^2+^/CaMKII/CREB Pathway

**DOI:** 10.1155/2021/3401654

**Published:** 2021-09-24

**Authors:** Guopeng Ding, Dandan Li, Yingjie Sun, Keyan Chen, Dandan Song

**Affiliations:** ^1^Postgraduate Training Base of Jinzhou Medical University in The General Hospital of Northern Theater Command, Jinzhou, Liaoning 121013, China; ^2^Department of Anesthesia, The General Hospital of Northern Theater Command, Shenyang, Liaoning 110016, China; ^3^Department of Anesthesiology, People's Hospital of Zhengzhou, Zhengzhou, Henan 450002, China; ^4^Department of Laboratory Animal Science, China Medical University, Shenyang, Liaoning 110122, China

## Abstract

**Objective:**

Cardiopulmonary bypass (CPB) is an important cardiac operation and also a high-risk procedure, leading to postoperative neurocognitive disorder. However, there are few effective drugs to treat the aftermath of CPB. Therefore, we observe the effect of kappa opioid receptor (KOR) agonist on cognitive disorders of rats after cardiopulmonary bypass (CPB) and investigate the mechanism of the Ca^2+^/calmodulin-dependent protein kinase (CaMKII)/cAMP responsive element-binding protein (CREB) pathway.

**Methods:**

A total of 40 Sprague Dawley rats were randomly divided into the sham operation group (sham group, *n* = 10), CPB model group (CPB group, *n* = 10), CPB + KOR agonist U50488H group (UH group, *n* = 10), and CPB + specific CaMKII antagonist + U50488H group (CKU group, *n* = 10). The changes in the rats' cognitive function were evaluated using the Morris water maze, the hippocampal histopathological changes were observed via hematoxylin-eosin (H&E) staining, and the apoptosis rate of neuronal cells was detected through terminal deoxynucleotidyl transferase-mediated dUTP nick-end labeling (TUNEL) staining. Moreover, enzyme-linked immunosorbent assay (ELISA) was applied to examine the changes in brain injury markers, inflammatory factors, and oxidative stress factors. The hippocampal variations in Ca^2+^ concentration and oxidative stress index (ROS) levels were measured by immunofluorescence staining, and western blotting was performed to determine the expression changes in the Ca^2+^/CaMKII/CREB pathway.

**Results:**

The KOR agonist could shorten latency, increase the swimming distance and residence time in the target quadrant, and ameliorate postoperative neurocognitive disorder (PND). Meanwhile, the KOR agonist relieved CPB-induced hippocampal and oxidative stress injuries, reduced NSE and S-100*β* expression, decreased the apoptosis rate, and repressed the inflammatory response, which alleviated the brain injury. In addition, U50488H was able to decrease Ca^2+^ influx and glutamate (Glu) level, inhibit *N*-methyl-D-aspartate receptor (NMDAR) expression, upregulate CaMKII expression, promote CREB phosphorylation, and increase the brain-derived neurotrophic factor (BDNF) level in CPB rats. However, the protective effects of KORs against PND were suppressed following the application of the CaMKII-specific antagonist.

**Conclusion:**

The KOR agonist activates the Ca^2+^/CaMKII/CREB pathway, which improves the brain injury and relieves PND in CPB rats.

## 1. Introduction

Cardiopulmonary bypass (CPB) is mainly applied in cardiac operations for ischemic, valvular, and congenital heart diseases, and aortic dissection [1]. However, its application in central nervous system complications after CPB has attracted more attention. Unfortunately, postoperative neurocognitive disorder (PND) has become one of the leading causes of disability and death of patients after cardiac operation under CPB [2]. According to reports, the incidence rate of a short-term cognitive disorder, in the first week after CPB, is as high as 40–60%, and a long-term neurocognitive disorder was reported to occur in 25% of the patients, which seriously affects their daily behavioral ability [3, 4]. Therefore, seeking for efficacious prevention and treatment measures, which tackle these issues at the source of pathogenesis, is of an important clinical significance in improving the incidence of PND and reducing death rate.

Neuroinflammation, especially inflammation in the hippocampal tissues, is a major reason of PND onset [5]. Both aged rats and mice manifest significant memory and learning deficits that are accompanied with the activation of microglial cells and increase in tumor necrosis factor-alpha (TNF-*α*) and interleukin (IL)-1*β* expressions in the hippocampus, resulting in nerve cell apoptosis and reduced learning and memory abilities [6, 7]. Moreover, the Ca^2+^/calmodulin-dependent protein kinase (CaMKII)/cAMP responsive element-binding protein (CREB) pathway plays vital roles in learning and memory [8]. Specifically, when abnormalities occur in the cognitive functions of the brain, glutamate (Glu) in hippocampal neurons rises, *N*-methyl-D-aspartate receptor (NMDAR) is overactivated, the Ca^2+^ cell membrane permeability increases, and the massive Ca^2+^ influx leads to cellular calcium overload. Furthermore, Ca^2+^ binds to CaMKII and activate CREB, which phosphorylation (p-CREB) regulates learning and memory abilities, by modulating the transcription and translation of genes that are related to learning, memory, and neuroprotection, and therefore participate in processes such as synaptic plasticity, long-term potentiation, and cerebral protection [9]. Hence, decreasing the release of neuroinflammatory factors, in the hippocampus and restraining Ca^2+^ influx, has crucial clinical significance in improving brain injury and in preventing and treating PND, caused by cardiac operation under CPB.

Kappa opioid receptors (KORs) are abundantly expressed in prefrontal cortex and other brain regions, which alleviate brain tissue injury and facilitate functional recovery in animal models and local cerebral ischemia [10]. Studies have demonstrated that KOR agonist U50488H can ameliorate the cognitive decline triggered by cholinergic dysfunction in mice, particularly during scopolamine-induced cognitive impairment [11]. The function is correlated with the cholinergic system and can be reversed by nor-BNI, a selective KOR antagonist. KORs are expected to become one of the treatment methods for mitigating PND, caused by cardiac operation under CPB. In this study, the CPB rat model was established and treated with KOR agonist to investigate the effect of the KOR agonist on the cognitive function and hippocampal neuronal injury and to explore the mechanism of action of the Ca^2+^/CaMKII/CREB pathway.

## 2. Materials and Methods

### 2.1. Laboratory Animals and Grouping

Sprague Dawley rats were purchased for CPB animal model preparation. A total of 40 SPF-grade male Sprague Dawley rats weighing 350–450 g [Laboratory Animal Using License No. SYXK (Military) 20120007 and Laboratory Animal Production License No. SCXK (Military) 20120006] were provided by the Department of Laboratory Animal of General Hospital of Northern Theater Command. All rats were randomly divided into 4 groups: sham operation group (sham group, *n* = 10), CPB model group (CPB group, *n* = 10), CPB + KOR agonist U50488H group (UH group, *n* = 10), and CPB + specific CaMKII antagonist + U50488H group (CKU group, *n* = 10). The present study was reviewed and approved by the Laboratory Animal Ethics Committee of General Hospital of Northern Theater Command.

### 2.2. Establishment of the CPB Model

The rats were anesthetized by intraperitoneal injection of 30 mg/kg pentobarbital sodium, fixed on an operation table in the supine position, subjected to tracheal intubation, and connected to a rodent ventilator and an anesthesia machine. The anesthesia was maintained by 2% isoflurane. A 24 G trocar was placed into the right femoral vein to open the venous access, from which 6% hydroxyethyl starch was infused at 0.5 mL/h. Later, a 22 G trocar was inserted into the left femoral artery to monitor real-time arterial pressure. Besides, a 22 G trocar was used for caudal artery puncture and an 18 G trocar, with an opening on the side of headend, was used for catheterization of the right jugular vein to accomplish CPB. After circuits' connection and fixation, the venous blood was drained into a blood reservoir and then reinfused into the body via the caudal artery following bypass in a peristaltic pump and oxygenation in an oxygenator. The medication was adjusted based on blood gas analysis and the following parameters were maintained: MAP >60 mmHg, pH in normal range, PaCO_2_ at 35–45 mmHg, and BE at −3–3 mmol/L. The bypass was gradually stopped when the hematocrit was higher than 0.25, the mechanical ventilation was restored. Subsequently, the circuits were removed, the mechanical ventilation continued, and the residual blood in the blood reservoir was slowly infused to sustain a stable circulation. If the rats were still alive 6 h after the bypass, the model would be successfully established. The rats in the UH group were intravenously injected with U50488H (1.5 mg/kg) 30 min before CPB. In the CK group, 5 *μ*L of the specific CaMKII antagonist KN93 (10 *μ*M) was injected into the lateral ventricle 60 min before CPB, and U50488H was injected 30 min later.

### 2.3. Morris Water Maze

The rat's cognitive function was accessed by Morris water maze. Three days after operation, the water maze test was performed for each group to observe the changes in behavioral and cognitive functions. The laboratory rats were put into water facing the pool wall from any quadrant and allowed to freely swim for 90s to find the hidden platform. The time of finding the hidden platform in the pool was recorded as the escape latency. The rats were tested for 5 consecutive days, the former 4 days of test were regarded as training periods, and the test results on the 5th day was taken as the spatial learning and memory performance. At 24 h after the hidden platform test, the platform was withdrawn. Next, rats were placed into water, from the same water entry point, and swimming path and allowed to swim for 60 s. The residence time in the original platform quadrant and times of crossing the original platform were recorded. Finally, the data were processed by a Morris water maze video analysis system.

### 2.4. Sample Collection

After the water maze test, rats in each group were anesthetized by isoflurane and then sacrificed by exsanguinations from the abdominal aorta. The blood was centrifuged to collect the serum, which was cryopreserved for later use. The brain tissues were isolated, parts were fixed in 4% paraformaldehyde, and the parts were stored in a freezer at −80°C.

### 2.5. Hematoxylin-Eosin (HE) Staining

The hippocampal histopathological changes were observed via hematoxylin-eosin (H&E) staining. The paraformaldehyde fixed brain tissues were placed in 70%, 80%, 90%, 95%, and 100% alcohol, transparentized by xylene, immersed in paraffin to prepare paraffin-embedded blocks and sliced to 4*μ*m-thick sections using a microtome. The sections were deparaffinized, stained with hematoxylin for 5 min, washed with phosphate-buffered saline (PBS), and differentiated with 1% hydrochloric acid alcohol. Next, the sections were stained with eosin solution for 30 s, dehydrated in gradient alcohol, and cleared and mounted in neutral balsam. Finally, the sections were observed under a light microscope and photographed (CX33, Olympus Corporation, Japan).

### 2.6. TUNEL Staining

The apoptosis rate of neuronal cells was detected through TUNEL. TUNEL assay kit (Roche Diagnostics, Mannheim, Germany) was employed to detect hippocampal neurons apoptosis and according to the manufacturer' instructions. The paraffin-embedded hippocampal tissues were cut into 5*μ*m-thick sections, processed with 50 *μ*L of TUNEL reaction solution, and incubated at 37°C for 60 min in the dark. This step was followed by the addition of 50 *μ*L of streptavidin-horseradish peroxidase (HRP) working solution onto the sections for incubation in a lightproof box for 30 min. Then, the nuclei were subjected to fluorescence staining using 4′,6-diamidino-2-phenylindole (DAPI) staining solution, and the sections were dehydrated, mounted in antifade fluorescence mounting medium, and photographed under a fluorescence microscope.

### 2.7. Enzyme-Linked Immunosorbent Assay (ELISA)

The brain injury markers, inflammatory factors, and oxidative stress factors were detected by ELISA assay. The protein expression levels of S-100*β* (SEA567Ra, USCN), the neuron-specific enolase (NSE) (SEA537Ra, USCN), and Glu (CES122Ge, USCN) in rat hippocampus; the levels of the inflammatory factors IL-1*β* (CSB-E08055r, CUSABIO), IL-6 (SEA079Ra, USCN), and TNF-*α* (SEA133Si, USCN) in the serum; and the oxidative stress indexes superoxide dismutase (SOD) (SES134Hu, USCN), malondialdehyde (MDA) (CEA597Ge, USCN), and glutathione peroxidase (GSH-Px) (CEA294Ge, USCN) were measured using ELISA kits and in accordance with the manufacturer's instructions. Specifically, 100 *μ*L of standard substances and 100 *μ*L of diluted samples were sequentially added into the wells of corresponding reaction plates and gently shaken for 30 s. Then, 100 *μ*L of serum samples was added into each well and incubated for 2 h at 37°C. Next, the plates were washed with PBST and 100 *μ*L of HRP-labeled secondary antibodies was added to each well and incubated for 30 min at 37°C. This step was followed by plate washing, the addition of 50 *μ*L of developer A and 50 *μ*L of developer B and color development in the dark for 15 min. After adding 50 *μ*L of stop buffer, the optical density (OD) value was read at 450 nm using a microplate reader (EXL800, USA). Finally, the standard curves were plotted with the OD value as the ordinate and the standard substance concentration as the abscissa, to obtain the curvilinear equation and *r* value. The concentration of the corresponding sample was calculated based on the curvilinear equation.

### 2.8. Immunofluorescence (IF)

The hippocampal changes in Ca^2+^ concentration and oxidative stress index (ROS) levels were measured by immunofluorescence staining. The paraffin-embedded hippocampal tissue sections were deparaffinized until rehydration, soaked in a 3% hydrogen peroxide solution, washed with PBS, and treated with 0.1 M sodium citrate for antigen retrieval. Subsequently, the sections were incubated in goat serum for 30 min at 37°C, a Ca^2+^ fluorescent probe, reactive oxygen species (ROS) probe, and brain-derived neurotrophic factor (BDNF) antibody (ab205067, Abcam, USA) were added and incubated again at 4°C overnight. After washing with PBS, the sections were incubated with fluorescence-labeled secondary antibodies for 30 min at 37°C and rinsed in PBS again. The nuclei were stained with DAPI and incubated at room temperature for 10 min, followed by washing with PBS, mounting in antifade fluorescence mounting medium, and photography under a fluorescence microscope.

### 2.9. Western Blotting

Western blotting was performed to determine the expression changes in the Ca^2+^/CaMKII/CREB pathway. The cryopreserved hippocampal tissues were added with 1 mL of protein lysis buffer containing 1% protease, homogenized, placed on ice for 30 min, and centrifuged at 12,000 rpm for 15 min at 4°C. The supernatants were collected, and their protein concentration determined by the bicinchoninic acid (BCA) method. Next, the proteins were subjected to sodium dodecyl sulfate polyacrylamide gel electrophoresis (SDS‐PAGE), transferred onto a membrane and sealed in skim milk for 2 h, followed by incubation with nuclear factor-kappa B (NF-*κ*B) p65 antibody (ab16502, Abcam, USA), B-cell lymphoma-2 (Bc1-2) (ab59348, Abcam, USA), Bcl-2-associated X protein (Bax) (ab32503, Abcam, USA), NMDAR2B antibody (ab65783, Abcam, USA), CaMKII (ab22609, Abcam, USA), CREB (ab32515, Abcam, USA), p-CREB (ab32096, Abcam, USA), BDNF (ab108319, Abcam, USA), and GAPDH antibody (ab181602, Abcam, USA) at 37°C for 1 h and at 4°C overnight. The membrane was washed 3 times with TBST for 10 min and then incubated with an HRP-labeled goat anti-rabbit IgG antibody for 1 h at 37°C. After membrane washing, the proteins were reveled using ECL kit and gel imaging system, and the absorbance was analyzed by Image Tools software.

### 2.10. Statistical Analysis

The SPSS 20.0 software was used for analysis and the experimental data were presented as mean ± standard deviation (*χ* ± *s*). A one-way variance analysis was utilized for comparing data between groups. *P* < 0.05 suggested that the difference was statistically significant.

## 3. Results

### 3.1. KOR Agonist Ameliorated Brain Injury and Alleviated PND in CPB Rats

The water maze test was applied to determine the cognitive function of the rats. In the hidden platform training, the latency of finding the platform was prolonged, and the swimming distance and residence time in the target quadrant were markedly decreased in the CPB group (vs. Sham group, *P* < 0.05). However, the KOR agonist U50488H could shorten the latency, increase the swimming distance and extend the residence time in the target quadrant (vs. CPB group, *P* < 0.05) (Figure 1(a)). The histopathological changes in the hippocampus were observed by H&E staining, and the results indicated that the CPB group had severe hippocampus injury, disorderly arranged cells, and a gradual widening of the intercellular space. However, the hippocampus injury was alleviated in UH group (Figure 1(b)). To clarify the state of rats' brain injury, the concentration of the brain injury markers was detected through ELISA. It was observed that the concentrations of NSE and S-100*β* were raised in the CPB group (vs. Sham group, *P* < 0.05)), while they were remarkably lower in the UH group compared to those in the CPB group (*P* < 0.05). These results suggest that the KOR agonist can ameliorate brain injury and alleviate PND in CPB rats.

### 3.2. KOR Agonist Inhibited Inflammation and Oxidative Stress Response in CPB Rats

The inflammatory response and oxidative stress injury in brain tissues are the main factors of CPB-induced PND; therefore, changes in inflammatory and oxidative stress factors in rats' sera and in each group were examined using ELISA. The results showed an increase in the serum concentrations of IL-1*β*, IL-6, and TNF-*α* (vs. Sham group, *P* < 0.05) (Figure 2(a)). In the UH group, the serum concentrations of inflammatory factors declined, and the expression of NF-*κ*B in the hippocampal tissues was repressed (Figure 2(b)), implying that KOR agonist can inhibit the CPB-induced inflammatory response.

The activated inflammatory response can facilitate oxidative stress injury, and ROS increase has been proved in neurodegenerative disorders. In this study, ELISA was first conducted to measure SOD, MDA, and GSH-Px serum contents, and the results showed that the KOR agonist could enhance the release of SOD and GSH-Px and suppress MDA (vs. CPB group, *P* < 0.05) (Figure 2(c)). Furthermore, IF was utilized to assess ROS expression in the hippocampus and demonstrated that ROS expression was raised in the CPB group and reduced in the UH group (Figure 2(d)), indicating that the KOR agonist can mitigate oxidative stress injury in CPB rats.

### 3.3. KOR Agonist Inhibited Hippocampal Neurons' Apoptosis in CPB Rats

The CPB-induced PND caused brain injury in rats, increased the expression of the pro-apoptotic factor Bax and decreased the expression of the antiapoptotic factor Bcl-2 (Figure 3(a)). According to the hippocampal neurons TUNEL staining results (Figure 3(b)), the apoptotic rate of the neuronal cells was notably lowered in UH group (vs. CPB group, *P* < 0.05) (Figure 3(c)), suggesting that the KOR agonist can inhibit neuronal apoptosis in CPB rats.

### 3.4. KOR Agonist Activated the Ca^2+^/CaMKII/CREB Pathway in CPB Rats

Under inflammation and oxidative stress stimulation, CPB could elevate Glu level in hippocampal neurons (Figure 4(a)), overactivate NMDAR (Figure 4(b)), increase Ca^2+^ cell membrane permeability, and stimulate massive Ca^2+^ influx, causing calcium overload in cells (Figure 4(c)). Furthermore, calcium plays a crucial role in nerve growth and synaptic remodeling. It binds to CaMKII to weaken CREB phosphorylation (Figure 4(d)), decrease BDNF level, and affect the brain learning and memory abilities. However, the KOR agonist was able to decrease Ca^2+^ influx and Glu level, inhibit NMDAR expression, promote CREB phosphorylation, and upregulate BDNF in CPB rats, thereby relieving the brain injury and mitigating PND in CPB rats.

### 3.5. KOR Agonist Ameliorated PND through the Ca^2+^/CaMKII/CREB Pathway

To further investigate the regulatory mechanism of the Ca^2+^/CaMKII/CREB pathway in the CPB model, the rats were administered with the CaMKII antagonist KN93, before CPB modeling, and then injected with the KOR agonist to observe the influence on PND in CPB rats. It was observed that the CKU group had increased levels of S-100*β*, NSE, and Glu (Figure 5(a)), increased apoptosis rate (Figure 5(b)), and a downregulated BDNF expression (Figure 5(c)). Besides, the latency of finding the platform was extended, but the swimming distance and residence time, in the target quadrant, were distinctly reduced (vs. UH group, *P* < 0.05) (Figure 5(d)).

## 4. Discussion

After a cardiac operation, PND is a common complication which can result in short-term negative effects, such as prolonging ICU length and hospitalization, increasing the incidence rate of perioperative complications and mortality rate, and attenuating the daily living activity [12]. In the long term, it reduces the quality of life and even increases the long-term mortality rate. During CPB, low perfusion or mean arterial pressure, unstable hemodynamics, cerebral thrombosis, systemic inflammatory response, anemia, hyperglycemia, and CBP trauma of CPB lead to neurocognitive decline after operation [13]. In the present study, the CPB rat model was established and treated with a KOR agonist, and its impacts on cognitive function, inflammatory response, oxidative stress injury and cell apoptosis were investigated. The results illustrated that the KOR agonist could alleviate the brain injury and relieve PND in CPB rats. The mechanism of action is associated with the activation of the Ca^2+^/CaMKII/CREB signaling pathway.

As a superfamily of G protein-coupled receptors, opioid receptors are mainly classified into three subtypes: *µ*-opioid receptors, KORs, and *δ*-opioid receptors. Although *µ*-opioid receptors are always the major targets of opioid analgesics, KORs are the most abundant opioid receptors in the human brain and serve as critical regulators in several physiological systems, including pain modulation, motor function, stress response, and emotional control [14]. A study elaborated that KORs can prominently relieve hippocampus injury, cognitive disorder, and learning and memory impairment triggered by ischemia [15]. U50488H is highly selective to *κ* site but has lower affinity to *µ*- and *δ*-opioid receptors. Besides, it can reduce damage to the hippocampal cortical area 1 (CA1) and ameliorate learning and memory deficits; thus, U50488H is extensively applied in research on the physiological effects of KORs.

The elevated levels of C-reactive protein and IL-6, in patients with senescence, senile dementia, and coronary artery grafting, are closely correlated with cognitive disorders. Using animal model studies, Cibelli et al. reported that systemic and hippocampal inflammations have intimate relations with the TNF-*α*, IL-1*β*, and NF-*κ*B pathways [16, 17]. It was revealed in these studies that U50488H could lower the serum levels of TNF-*α*, IL-1*β*, and IL-6, repress NF-*κ*B expression in the hippocampus, and reduce the apoptosis rate of hippocampal neurons in CPB rats, through the specific activation of KORs on hippocampal neurons. These results prove that U50488H can improve PND in CPB rats.

CaMKII is an important player in modulating synaptic plasticity and hippocampus-dependent learning and memory and is implicated in regulating neurotransmitters' synthesis, release, and signal transduction [18, 19]. Human cognitive learning disorders and vascular and various central nervous system diseases are accompanied with changes in CaMKII levels. Mice with CaMKII deficiency may manifest impairments in hippocampus-dependent spatial learning and memory. According to the results in this study, the Glu level was raised in the hippocampal neurons of CPB rat model. The activated NMDAR caused a calcium overload in the hippocampal neurons, a decrease of CaMKII expression, and a suppression of CREB phosphorylation. Moreover, p-CREB regulated learning and memory abilities by modulating the transcription and translation of genes related to learning, memory, and neuroprotection, which participate in synaptic plasticity. All the findings demonstrate that the incidence of PND after CPB is associated with the decline in memory protein expression.

Previous studies have demonstrated that KORs can negatively regulate *β*-adrenergic receptor via the PKC/cAMP pathway, the inositol 1,4,5-triphosphate (IP3)/Ca^2+^ pathway, and the receptor itself, thereby realizing myocardial protection [10, 20]. The IP3/Ca^2+^ pathway can further activate calmodulin and the downstream regulatory proteins CaMKII and CREB to regulate synaptic plasticity, form neurons, and maintain long-term memory. In this study, KORs could increase CaMKII expression, activate CREB phosphorylation, and upregulate BDNF expression in CPB rats. It has been confirmed that CREB and BDNF can ameliorate cognitive disorders, facilitate nerve cells growth and differentiation, and participate in the regulation of long-term synaptic plasticity [21]. This implies that the KOR agonist can activate the Ca^2+^/CaMKII/CREB pathway and promote nerve cells growth and differentiation in CPB rats. In addition, the effects of the CaMKII antagonist KN93 combined with U50488 on CPB were investigated to explore the regulatory mechanism of the Ca^2+^/CaMKII/CREB pathway. The results revealed that the protective effect of KORs against PND was inhibited, and that PND in CPB rats was aggravated after the application of the CaMKII-specific antagonist, suggesting that the KOR agonist can alleviate PND in CPB rats through the Ca^2+^/CaMKII/CREB pathway. However, the KOR agonist is involved in regulating cerebral protection in CPB rats via multiple pathways; therefore, whether it improves neurocognitive function in the perioperative period and protect the brain, by coordinating with the pathway, requires further investigations through in-depth studies.

## Figures and Tables

**Figure 1:** The KOR agonist ameliorated brain injury and alleviated PND in CPB rats. (a) Water maze test. (b) HE staining. (c) The brain injury markers detected by ELISA. ^∗^*P* < 0.05.

**Figure 2:** The KOR agonist inhibited inflammation and oxidative stress response in CPB rats. (a) Inflammatory factors detected by ELISA. (b) The expression of NF-*κ*B protein detected by western blot. (c) SOD, MDA, and GSH-Px serum contents detected by ELISA. (d) The expression of ROS detected by IF. ^∗^*P* < 0.05.

**Figure 3:** The KOR agonist inhibited hippocampal neurons' apoptosis in CPB rats. (a) The expression of Bax and Bcl-2 proteins detected by western blot. (b, c) TUNEL staining. ^∗^*P* < 0.05.

**Figure 4:** The KOR agonist activated the Ca^2+^/CaMKII/CREB pathway in CPB rats. (a) Glu level in hippocampal neurons detected by ELISA. (b) The expression of NMDAR protein detected by western blot. (c) The expression of Ca^2+^ detected by IF. (d) The expression of CaMKII, CREB, and BDNF proteins detected by western blot. ^∗^*P* < 0.05.

**Figure 5:** The KOR agonist ameliorated PND through the Ca^2+^/CaMKII/CREB pathway. (a) The brain injury markers and Glu level detected by ELISA. (b) TUNEL staining. (c) The expression of BDNF detected by IF. (d) Water maze test. ^∗^*P* < 0.05.

## Data Availability

The datasets used and analyzed during the current study are available from the corresponding author upon reasonable request.
